# Effect of Sandplay Therapy on the Mental Health Level of College Students

**DOI:** 10.1155/2022/3716849

**Published:** 2022-06-03

**Authors:** Gaoyong Li, Xue Wu

**Affiliations:** School of Economics Management, Kaili University, China

## Abstract

To analyze the effect of sandplay (SP) therapy on the mental health level of college students. 500 college students were openly recruited, using the University Student Mental Health Questionnaire (UPI) to screen out 76 students in the UPI category. 34 college students were randomly selected and divided into two groups, 17 in the control group and 17 in the SP therapy group (experimental group); the control group received no treatment, and the experimental group was treated with SP therapy, to analyze the differences between groups before and after the intervention of SCL-90 and self-made group self-reflection questionnaire. (1) With a detection rate of 15.2 percent, 76 of the 500 college students solicited openly were identified as UPI students; (2) except for the terror factor, there were significant differences in other aspects and overall scores for the experimental group following SP therapy intervention, and the scores reduced. There were no significant differences in the total scores and scores of all factors in the control group (*P* > 0.05). The overall score, somatization, interpersonal connection, depression, paranoia, and psychosis were all significantly different between the experimental and control groups in the independent sample *t*-test (*P* < 0.05).

## 1. Introduction

SP therapy is an approach where the study subjects freely choose toys from the toy rack in the company of the therapist. It is a form of psychotherapy in which one performs self-expression in a box of fine sand, which is also called sand table play therapy [1]. The treatment process of the box court consists of two main parts: the creation of the group box court and the discussion after creation. SP therapy advocates that in a safe and free space, the healer takes the “motherly role” of a mother and child, faces the visitor with a silent, empathic, and understanding witness attitude, and emphasizes and believes in “self-healing power” [2, 3]. For a long time, intervention studies of SP therapy have focused on case studies [4]. The materials for SP therapy include a 57 × 72 × 7 (cm) sandboxes (painted blue on the inside), sand, and various types of toy models [5]. Its treatment hypothesis believes that everyone has a tendency to heal their psychological trauma in the depths of their souls, if there is a “free and protected” space; the self-healing ability of research subjects can be brought into play [6]. In the mental health education of college students, the application of individual court and group court should be combined to make full use of its nonverbal advantages in the court therapy [7], to help students express their emotions well in the early stages of adult development, to provide a good solution for students who have problems in learning burnout, social anxiety, maladjustment, career decision-making, and so on, and to encourage them to constantly improve their ability of self-exploration, constantly explore the unknown self, and promote the improvement of self-healing ability and the growth of healthy psychology [8, 9]. Negative emotions can be channeled, psychological trauma can be cured, self-awareness can be enhanced, and self-potential can be stimulated when college students can freely express their ideas and therapists can make college students feel accepted, understood, and included through noncritical communication [10, 11]. 500 college students were openly recruited, using the University Student Mental Health Questionnaire (UPI) to screen out 76 students in the UPI category; 34 college students were randomly selected and divided into two groups, 17 in the control group and 17 in the SP therapy group (experimental group), and the experimental group was treated with SP therapy.

SP therapy for college students is essentially an encouraging and reeducation procedure. Its main purpose is to foster college students' social interests. It has three primary functions: self-healing ability, way of life, and the spirit of mental health education for college students including diagnosis and assessment, expression, and communication.

The arrangements of the paper are as follows:

Section 2 discusses the materials and methods.  Section 3 analyzes the results.  Section 4 examines the discussion.  Section 5 concludes the article.

## 2. Materials and Methods

Here, we discuss the general information and evaluate the various methods. We examine the observational index and analyze the statistical method.

### 2.1. General Information

500 college students were openly recruited, using the University Student Mental Health Questionnaire (UPI) to screen out 76 students in the UPI category; 34 college students were randomly selected and divided into two groups, 17 in the control group and 17 in the SP therapy group (experimental group). There was no significant difference in general data between the two groups (*P* > 0.05).

### 2.2. Methods

The control group received no treatment, the experimental group was treated with SP therapy, and the details were as follows.

1. The sandbox: a sandbox contained half a box of sand, measuring 57 cm in length, 72 cm in width, and 7 cm in height, painted blue on the inside and dark or woody on the outside
2. The sand tools: SP therapy requires a wide variety of toys
3. The implementation process: each group would make a group box court once a week, 5 to 6 rounds each time, and the time would be about 1.5 to 2 hours. Each time, the order of production was determined according to the drawing, punching, or custom form; intervention was given to the experimental group during each production—or according to the main research content of positive psychology, the theme (college life, class, and home) was designated before the production. Or in the production direction, sand movement and discussion and sharing in combination with Baker reconstruction of core belief technology and Ellis rational emotional therapy were conducted to give guidance [12]. For the recording of sand table works, different consultants also had different practices. Individual sand table records were utilized by some consultants to record which sand tools were placed by the research subjects and in what sequence, as well as the first and last sand tool and the number of animals and plants, humans, and structures. Some consultants took photos; some consultants used sketches or scribbled notes; there were consultants who combined a variety of records

### 2.3. Observational Index

To analyze the differences between groups before and after the intervention of SCL-90 and self-made group self-reflection questionnaire.

1. University Student Mental Health Questionnaire (UPI) [13]: UPI was one of the most widely used mental health status tests at present. There were a total of 60 questions, of which 4 questions were false questions and the remaining 56 questions were scored, with the highest score of 56; the minimum score was 0. The higher the total score, the lower the mental health level
2. Symptom Checklist 90 (SCL-90) [14]: the scale had a total of 90 items and was divided into 10 factors. Each factor reflected one aspect of the subject, respectively. The 10 factors were somatization, obsessiveness, interpersonal relationship, depression, anxiety, hostility, fear, paranoia, psychosis, and others (mainly reflecting sleep and eating). A 1- to 5-point scoring system was used for each of the five grades. From 1 point for asymptomatic to 5 points for severe symptoms, the total score was the sum of the scores of 90 items. The lower the score, the better the psychological condition of the subject

### 2.4. Statistical Method

The statistical software SPSS 23.0 was used for analysis. The *t*-test was used for comparison data between groups, and the *χ*^2^ test was used for counting data. *P* < 0.05 was considered to be statistically significant.

## 3. Results

### 3.1. Result of UPI

Of the 500 college students recruited publicly, 76 were detected as UPI students, with a detection rate of 15.2%. 34 college students were randomly selected. Result of UPI is shown in Table 1.

### 3.2. Result Symptom Self-Evaluation

For the experimental group, after the intervention of SP therapy, there were significant differences in other factors and total scores except the terror factor, and the scores decreased. There were no significant differences in the total scores and scores of all factors in the control group (*P* > 0.05). The independent sample *t*-test of the posttest data between the experimental group and the control group showed significant differences in total score, somatization, interpersonal relationship, depression, paranoia, and psychosis (*P* < 0.05). Result symptom self-evaluation is shown in Table 2.

## 4. Discussion

SP therapy is a therapy coming from Adler School that instructs group members to work together to produce a work that reflects a theme and to evaluate it effectively [15]; Adler style-guided chamber therapy from the perspective of Adler School attaches importance to the final fictional goal of the client and the activity towards that goal and believes that once the client undergoes changes in the experience, it is likely to transfer them to real life [16]. The nonverbal creation stage at the beginning of SP therapy avoids the pressure of direct face-to-face communication and effectively helps individuals with low psychological resilience to express themselves, which can maximize not being subject to the control of other people's words, the true expression of their own, figuring out other people's mind, and their own thoughts to match the thoughts of others [17, 18]. The essence of SP therapy for college students is a process of encouragement and reeducation. Its basic goal is to cultivate the social interests of college students. It has three key roles: sousing self-healing ability, life style diagnosis, and assessment; expression and communication are exactly in line with the spirit of college students' mental health education: promoting students' all-round development and preventing psychological development defects [19, 20]. The creation and discussion process of the box court makes the group members express themselves effectively as much as possible. The collision of each student's experience will produce new experience, which will be integrated into the group members' own experience, and the new construction will come into being [21]. The whole intervention process of SP therapy is easy to trigger the inner experience of college students and imperceptibly learn interpersonal skills [22]. Due to various reasons, college students have a certain weariness, inferiority, not strong self-restraint ability, behavioral problems, and prominent problems; it is of great significance to strengthen and improve the construction of big heart curriculum for promoting students' overall and healthy development and enhancing the effect of mental health education [23]. In line with the “student-centered” education and teaching philosophy, with teachers as guides and organizers, let students as learners and experiencers learn in experience, feel in learning, and grow up healthy in perception [24].

This study showed that (1) of the 500 college students recruited publicly, 76 were detected as UPI students, with a detection rate of 15.2%; (2) except for the terror component, there were significant variations in other factors and overall scores for the experimental group following the intervention of SP therapy, and the scores reduced. In the control group, there were no significant differences in total scores or scores for all criteria (*P* > 0.05). The overall score, somatization, interpersonal connection, depression, paranoia, and psychosis were all significantly different between the experimental and control groups in the independent sample *t*-test (*P* < 0.05).

## 5. Conclusion

SP therapy was an effective method to improve the mental health of college students.

## Figures and Tables

**Table 1:** Result of UPI.

Groups	Preintervention category	Postintervention category	Intervention efficiency
Control group (*n* = 17)	17	17	No intervention
Experimental group (*n* = 17)	17	2	88.24%
*χ* ^2^			26.842
*P*			<0.05

**Table 2:** Result symptom self-evaluation.

Factors	Pretest		Posttest		t1①-②	t2②-④	t3④-③	t4①-③
	Experimental group	Control group	Experimental group	Control group				
Total scores	201.0 ± 34.2	190.1 ± 43.2	167.8 ± 36.6	182.0 ± 45.3	0.9	0.9	2.2^∗^	4.1^∗∗^
Somatization	19.8 ± 4.1	20.0 ± 6.3	16.6 ± 4.4	19.5 ± 6.8	-0.02	0.6	2.0^∗^	3.4^∗∗^
Obsessiveness	25.5 ± 7.0	25.1 ± 6.1	22.8 ± 6.0	25.0 ± 6.0	-0.05	0.3	1.1	2.3^∗^
Interpersonal relationship	22.1 ± 4.6	20.8 ± 5.6	18.5 ± 4.4	20.5 ± 6.2	1.4	0.4	2.0^∗^	2.8^∗∗^
Depression	29.1 ± 7.6	26.4 ± 7.0	23.0 ± 6.0	25.5 ± 8.5	2.0	0.5	2.1^∗^	3.8^∗∗^
Anxiety	22.1 ± 5.2	21.4 ± 6.4	19.4 ± 4.6	20.8 ± 6.4	0.2	0.7	1.1	2.6^∗^
Hostility	12.6 ± 3.5	11.3 ± 3.0	10.3 ± 3.1	10.6 ± 3.2	1.8	1.3	1.0	2.4^∗^
Fear	15.8 ± 9.1	16.5 ± 5.2	12.7 ± 3.5	12.8 ± 8.4	0.3	1.6	1.3	1.3
Paranoia	13.7 ± 3.3	11.6 ± 3.5	10.9 ± 3.3	11.8 ± 4.3	5.2	-0.4	3.2^∗∗^	4.6^∗∗^
Psychosis	20.3 ± 5.6	19.6 ± 6.2	17.0 ± 4.3	18.0 ± 5.1	0.3	1.5	1.2	3.5^∗∗^
Others	15.3 ± 3.1	13.2 ± 3.5	12.1 ± 6.4	12.3 ± 4.2	2.2	1.0	3.1	1.2

Note: ^∗^*P* < 0.05, ^∗∗^*P* < 0.01.

## Data Availability

The data used to support the findings of this study are included within the article.
